# An Empirical Study on the Influence of College Students' Physical Fitness on the Level of Public Health

**DOI:** 10.1155/2022/8197903

**Published:** 2022-10-05

**Authors:** Yinghong Zhang

**Affiliations:** Harbin University, Harbin 150086, China

## Abstract

As a compulsory course in universities, physical fitness is an important part of public health. At present, research on physical fitness lacks a comprehensive evaluation method, which cannot accurately guide public health. Based on this, this paper compares the key factors affecting public health, aiming to better guide public health and improve the level of public health. In this paper, 219 college students were selected as the research object, using statistical analysis methods, to find out the significant differences in influencing factors. Then, regression analysis is carried out on different influencing factors to determine the key factors affecting physical fitness. The results show that physical fitness level, exercise frequency, and physical injury are the key factors affecting physical fitness and have a serious impact on public health, with an impact level of about 70~80%. Therefore, colleges and sports departments should set out from the above factors, formulate a development plan for physical fitness, and promote the improvement of public health.

## 1. Introduction

At present, the prevention and control of the COVID-19 epidemic have become normalized. Although the COVID-19 epidemic has had a huge impact on the national economy, culture, education, etc., it has also “strongly” improved the health literacy of the whole people. Due to the impact of the epidemic, the public's awareness of health has been greatly enhanced, and more emphasis has been placed on fitness exercise and healthy culture. The Ministry of Sports attaches great importance to the development of physical injury and physical fitness and regards it as the main driving factor to improve the public health level and to promote the improvement of the public health level. However, physical fitness needs correct guidance to play a role in promoting public health [1]. Some scholars believe that physical fitness should integrate various factors, such as physical fitness level, fitness awareness guidance level, exercise frequency, and physical injury; otherwise, it is difficult to play its role [2].

## 2. Literature Review

The study on college students' physical fitness influences domestic public health level. Some scholars believe that physical fitness needs a certain method as the basis and integrates with the sports connotation to give full play to its comprehensive advantages [3]. Studies have shown that college students' physical fitness has a significant impact on public health, but the degree of impact is not clear. Some scholars believe that the effective development of college students' physical fitness activities will promote public health development. Therefore, the impact of college students' physical fitness activities on public health will be the future research direction and research hotspot. Therefore, it is of great significance to strengthen the research on college students' physical fitness and analyze the influence on public health. At present, there are some controversies in the research of physical fitness, and there is also a lack of effective methods as guidance [4]. Therefore, it is an urgent problem for relevant experts to verify the effectiveness of physical fitness and its role in improving public health. The specific investigation needs are shown in Figure 1.

According to the survey in Figure 1, the average demand for physical fitness changes by 32%, and the actual demand for public health to affect the value is rising, and the difference between them is increasing year by year [5]. In 2020 and 2020, the demand for improving the impact value of public health level is reasonable, and the demand for physical fitness fluctuates greatly in 2018 and 2019, which further shows that physical fitness cannot meet the impact value demand of public health level, and further research will be carried out in the future. From the above analysis, we can see that there are many empirical studies on college students' physical health abroad, while there are many theoretical studies in China, lacking practical case analysis. At the same time, there is an increasing demand for college students' physical health in China, but there are relatively few actual case studies. Therefore, the physical health of college students is the focus of future research, and case analysis will be the focus of research. Therefore, there is a big gap between domestic and foreign research on college students' physical health. Based on the above reasons, this paper analyzes the influence value of physical fitness on the public health level under the background of the COVID-19 pandemic and finds out the factors affecting the value of the public health level [6].

## 3. Method

### 3.1. Mathematical Analysis of Related Problems

Suppose 1: The public health level is *T* composed of any public health indicators *x*_*i*_, which is expressed as *T* = {*x*_1_, ⋯*x*_*n*_}: the COVID-19 pandemic background is *K*, the influence ratio of physical fitness is *c*, the fitness time is *t*, and the value is *v*, then the effect of physical construction on public health level is shown in Formula (1).

(1) $$\begin{array}{c} T=\prod K\left|\underset{t,i}{\sum }\frac{t.c}{v}x_{i}+\xi .\right. \end{array}$$

Among them, *ξ* is the sports health adjustment policy under the COVID-19 pandemic. Because this paper is a periodic regional survey, the analysis of relevant parameter data is fixed, and the data sources are statistical yearbooks and local public health data [7].

**Hypothesis 1 .**

The time of physical fitness is *w*, the age of the exerciser is *O*, the probability of disease is *p*, and the degree of value influence is *F*, then the public health impact value is shown in Formula (2).

(2) $$\begin{array}{c} F=\cdot \underset{w}{\prod }\frac{O\cdot T}{D\cdot p}. \end{array}$$

Among them, *F* is a numerical variable, which should be accurate to 0.001 [8].

**Assumption 1 .**

The improvement rate affecting the value level is *H*, and the exercise effect is *B*: physical fitness level, fitness consciousness guidance level, exercise frequency, and the proportion of physical injury *c*_*i*_/*C*, and the exercise effect is divided into five grades, each of which is 20%, then the improvement rate affecting the value level is calculated as shown in Formula (3).

(3) $$\begin{array}{c} H=B\cdot \frac{\sum_{i}c_{i}}{C}+\xi . \end{array}$$

According to Formula (1)-(3), the overall analysis of public health levels is carried out. Hypothesis 4: The results of overall public health level are *P*: physical fitness level *P*_1_, physical injury is *P*_2_, fitness consciousness guidance level is *P*_3_ and exercise frequency is *P*_4_, and the corresponding tests are completed [9]. By comparing before and after the test, find out the key points and factors of existing problems and calculate the overall public health level as shown in Formula (4).

(4) $$\begin{array}{c} P=\prod \left(\frac{H}{\sum_{i=1}^{3}F_{i}}\right). \end{array}$$

### 3.2. Research Process of Public Health Level

According to the above analysis, the research process of the public health level is as follows, and the specific steps are as follows:

The first step, with the help of sports expert groups and authoritative organizations, is to carry out physical fitness from the perspectives of physical fitness level, fitness awareness guidance level, exercise frequency, physical injury, etc., and to investigate the influence value of public health level [10].

The second step is to score the impact value of public health level by experts with more than 2 years and its experience. At the same time, according to different investigators, provide corresponding physical fitness and finally make a comprehensive evaluation.

The third step is to analyze the data of public health level by SPSS21.0 software, express the counting data by %, and carry out the *X*^2^ test; $\bar{x}\pm s$ is used for measurement data, and the *T*-test is adopted to ensure the rationality of data [11]. The fourth step is to analyze the factors for improving public health and determine the improvement measures according to multiple regression analysis [12].

The fifth step is to output the output results of the public health level [13].

### 3.3. General Information of Public Health Surveyors

219 subjects, aged 13~56 years, with an average age of 43.21 ± 1.62 years, were selected as subjects. Impact value level: effective impact value is 16, invalid impact value is 4. The value influence degree is 2~6 grades, and the average value influence degree is 4.22 ± 1.03 grades. The index ranged from 3.11 to 3.45, with an average index of 6.13 ± 1.0. There is no significant difference in age, income, gender, and exercise time among the respondents, and they all sign the survey consent form, and the survey can be statistically analyzed with the consent of the Tourism Bureau of the Ministry of Sports [14]. The specific results are shown in Figure 2.

From the contents in Figure 2, it can be seen that the influence of college students' physical fitness on public health level is significantly better than that of physical fitness. Moreover, the change range of college students' physical fitness is small, which is significantly better than traditional fitness activities, indicating that the impact on public health level is relatively stable, further verifying the advantages of college students' physical fitness. Inclusion criteria are the following: (1) conforming to the evaluation criteria of public health level in the Guide to Public Health Level put forward by the Ministry of Education; (2) fill in less than 30 pieces of information [15]; (3) the investigator's exercise ability is normal, and there are no other related diseases; (4) the investigator cooperates with relevant research; (5) the investigator's bad reputation [16].

Exclusion criteria are as follows: (1) there are family genetic diseases [17]; (2) investigators have fractures and muscle strains [18]; (3) those with motor disorders; (4) those who quit halfway.

### 3.4. Questionnaire

According to Lu Jia and other scholars in 2001 who revised the “Public Health Survey Research” questionnaire, combined with the relevant literature at home and abroad, the questionnaire designed in this paper to ensure the rationality of questionnaire, to send this questionnaire to the university, and to revise the questionnaire. In this paper, 219 universities were selected as the research objects, and 219 questionnaires were distributed. The questionnaire recovery rate was 100%, and there were no questions left. All college students have signed a good faith agreement, and the writing problems are the actual situation. The questions in the questionnaire are based on the questionnaires such as the “College Students' Physical Fitness Standards” and “Public Health Level,” combined with the actual situation. At the same time, experts are hired to revise the contents of the questionnaire to ensure its validity of the questionnaire. At the same time, the questionnaire questions whose reliability and validity do not meet the requirements are eliminated to ensure the validity of the questions. Finally, the questionnaire is divided into four aspects, namely, audience basic information, physical fitness factors (reliability = 0.763, validity = 0.812), fitness awareness (reliability = 0.723, validity = 0.713), and overall health level (reliability = 0.791, validity = 0.743) [19]. There are 8 physical factors, each with 3 points. There are 6 questions about fitness awareness, each with 4 points. The overall health level consists of 8 questions, each with 4 points. The total score of the whole questionnaire is 100, and there are significant differences among the survey questions (*P* < 0.05).

### 3.5. Research Methods

The comparison of physical fitness level and fitness consciousness guidance level showed that there was no significant difference (*P* > 0.05), but physical fitness was significantly better than before implementation, and there was a significant difference (*P* < 0.05). After physical fitness, the level of physical fitness consciousness guidance in the general group was significantly better than that in the influence value group, with a significant difference (*P* < 0.05). The results are shown in Table 1.

From the data in Table 1, it can be seen that the public health level of the group carrying out physical fitness for college students has not changed before the implementation, but after the implementation of physical fitness, it is significantly higher than that of the group without physical fitness for college students. This data shows that the development of college students' physical fitness can promote the improvement of public health, and there is a significant correlation between them. The data in Table 2 shows that the public health level of the two groups has been greatly improved after the implementation of physical fitness for college students, which further proves that physical fitness can promote the public fitness level. Physical fitness level and fitness consciousness guidance are improved through physical fitness, which mainly reflects the role of physical fitness. By improving physical fitness, frequency, and awareness, and cooperating with other auxiliary means, physical fitness under the COVID-19 pandemic can be realized and has an impact on public health. The matching between physical fitness and public health level can improve the public health level and highlight the value of physical fitness. Exercise frequency, physical injury, and value influence range were compared. After physical fitness, in the exercise frequency of the general group, the influence range of physical injury and value is better than that of the influence value group, and there are significant differences (*P* < 0.05). The results are shown in Table 2.

Physical fitness plays an obvious role in public health level and has completed the improvement of public health level, which is liked by investigators. In the survey, it was found that 56% of the respondents did not implement physical fitness, and 32% of the respondents recommended physical fitness through friends. The problems in Table 3 are mainly that the investigators ignored the We Media platform and lacked the early publicity of physical fitness, resulting in an insufficient understanding of physical fitness. Physical fitness is a fitness activity according to the level and type of public health [20]. It can be seen from this that the investigators neglect physical fitness. However, there are some problems in physical fitness, such as a lack of investigation of target objects and target investigators in the early stage, which leads to poor understanding of physical fitness investigators. The overall result is shown in Figure 3.

From the fishbone diagram in Figure 3, it can be seen that weekly continuous fitness and regular physical training will improve the public health level. The effect of physical fitness on public health level is very significant, and the effect is significant, and the negative impact is relatively small. The results in Figure 3 suggest that regular and regular physical fitness for college students can not only improve their health level but also significantly impact public health. Multiple regressions of public health level affect the value. The general clinical data of the respondents and the evaluation elements with significant differences in Tables 1 and 2 are assigned by a single factor, and the results are shown in Table 3.

In the process of physical fitness, the investigators conducted muscle, strength, endurance, and other training. However, in the process of physical fitness, the investigators only carried out unilateral physical fitness, lacking relevant guidance. Some investigators could not deeply understand the role of physical fitness, which further reduced their awareness of investigators. Some investigators will confuse fitness and public health, which is not conducive to the implementation of physical fitness. Investigators generally believe that physical fitness is too complex and lacks personality, which will further raise ticket prices. On the whole, the complexity of physical fitness is higher than that of other fitness activities, so complexity is also an important factor of physical fitness. Logistic Cox analysis is carried out with research methods as independent variables and evaluation elements with significant differences as independent variables. The results are shown in Table 4.

It can be seen from Table 4 that physical fitness level, exercise frequency, physical injury, and value influence range are all evaluation factors of public health level influence value. Among them, physical health level, exercise frequency, and value range are the main factors affecting public health level, and training injuries are also the main factors affecting public health level. However, the awareness of fitness guidance is not the main factor affecting the level of public health, so we can ignore the related factors. In addition, the influence of value scope is the largest, followed by training frequency, training injury ranks third, and finally physical health level. Therefore, college students' physical fitness should start from the above factors and formulate corresponding measures to improve the influence of physical fitness on public health. The overall result is shown in Figure 4.

From the contents in Figure 4, it can be seen that the frequency of college students' physical fitness has an obvious influence on the level of public health, and there is a linear relationship between them. At the same time, the frequency of college students' physical fitness has an obvious influence on physical injury, and there is a linear relationship between them. Therefore, the frequency of college students' physical fitness has a linear relationship with the level of public health and physical injury. How to reduce the physical injury caused by physical fitness is a problem that needs to be solved in college physical education. The final result of physical fitness shows that after the physical fitness observation of all the respondents, one muscle strain occurred in the influencing value group. There was a significant difference in the incidence of complications among the respondents (*x*^2^ = 12.625).

## 4. Results and Discussion

### 4.1. Overview of the Impact Results of Public Health Level

Many factors, such as self-constitution, fitness awareness, and lack of effective guidance, will lead to unsatisfactory influence value of public health level [21]. The survey results show that the failure rate of public health level in China is 12.4%, and the ratio is increasing year by year. The results show the following: The sports items of the investigators have not been effectively implemented within 3 ~ 4 months, and the influence value will affect the graduation of the investigators and the improvement of their physical fitness. The key to the implementation of the public health level project is to improve muscle function and shorten nerve response time. Lack of scientific implementation guidance, it is easy to further affect the impact value of investigators, and their random implementation methods have a poor impact on the value. Therefore, accurately judging the implementation effect of physical fitness is the key to the improvement of public health levels and the focus of experts in the future.

### 4.2. Implementation Effect of Public Health

Under the background of the COVID-19 pandemic, this paper adopts the implementation method of physical fitness, and the results show that there is no significant difference between the implementation level of physical fitness and the guidance level of fitness consciousness, but there is a significant difference between the implementation level after physical fitness and the implementation level before physical fitness. After physical fitness, the general group's physical fitness level and fitness consciousness guidance level are significantly better than those of the influence value group, and there are significant differences. Therefore, in the context of the COVID-19 pandemic, physical fitness can accurately influence the value of expert sports guidance, find out the problems of physical fitness of investigators, improve the level of public health, and influence the value level. Among them, although the daily fitness implementation method is the main implementation means to improve the public health level project. There are some problems, such as unsatisfactory implementation effect, slow value promotion, and long value influence. Under the background of the COVID-19 pandemic, experts judge the fitness effect of investigators by their own experience, which not only is the scheme inaccurate but also has a certain impact on the physical and psychological of investigators in the process of affecting the value. In addition, the muscle strain and joint damage will affect the score of physical fitness level and exercise frequency or reduce the guidance level of fitness awareness and affect the value level. Under the background of the COVID-19 pandemic, in the post-implementation investigation, there was found that one muscle strain, one joint injury, and one illness occurred after one month of physical fitness. Two months after physical fitness, one person developed the local infection, but after the rest, the above symptoms all recovered, which indicates that physical fitness has a great positive impact on public health. According to some scholars' investigation, under the background of the COVID-19 pandemic, after the implementation of physical fitness, the scores of the physical fitness level of 45 respondents increased to 23.21~31.62 points, and the guiding level of fitness awareness increased to 14.19~21.14 ml, and the exercise frequency increased to 45.63~51.92, which was significantly better than the investigators who did not implement physical fitness and was consistent with the research results of this paper, further verifying the value of physical fitness on a public health level. Moreover, in the implementation of physical fitness, there was only 2 of the 45 respondents had joint redness, which was consistent with the results of this study [22].

### 4.3. Influencing Factors of Public Health Implementation Effect

In the survey, there are significant differences in the evaluation factors of single-factor analysis, exercise frequency, physical injury and value impact range, and physical level; exercise frequency is the impact of public health level of the value of the evaluation factors. Under the background of the COVID-19 pandemic, the OR of exercise frequency and physical injury are 2.424 and 2.103, which may be related to excessive exercise frequency, muscle strain, insufficient blood supply, decreased joint function, and other factors.

## 5. Conclusions

Physical fitness is an important part of college teaching, and it is also the basis for college students to improve their own quality. Based on the research on college students' physical fitness, this paper analyzes the influence on public health. Firstly, the general information about college students is collected and compared accordingly. Then, the differences of the indicators for comparative analysis found that there are significant differences in the influencing factors. Finally, regression analysis is carried out on relevant indicators to study the impact of indicators on public health. The results show the following:

This paper analyzes the impact on public health through research on the physique of college students and finds the main influencing factors. The results show the following: (1) There is no significant difference in the general data of college students, which can be compared statistically. (2) The matching degree of public health level, the intensity of publicity, the standard of investigators, the coherence, and complexity of sports are the main factors affecting the public health level, and the influence is very significant. (3) Universities should strengthen the analysis of the above indicators, formulate corresponding physical fitness programs, and promote college students to carry out physical fitness activities. (4) Universities should strengthen the publicity of physical fitness, encourage college students to pay attention to public health, hire famous domestic experts to give lectures, and increase the guidance of physical fitness. (5) The implementation of physical fitness can improve the level of public health, so it is necessary to strengthen college students' physical fitness. This study also has some limitations, mainly reflected in the collection of related data loss, data pretreatment not enough, and an increase in the error of research results. In addition, there are some deficiencies in this paper, such as the correlation between physical fitness level, exercise frequency, physical injury, and value influence range. For another example, before choosing the fitness research method, there is a lack of qualitative analysis of the above evaluation elements. In future research, we should focus on the analysis of the above aspects to improve the research depth of this topic.

## Figures and Tables

**Figure 1:** Relationship between physical fitness supply and public health level requirements.

**Figure 2:** Comparison of physical fitness among different groups.

**Figure 3:** Fishbone diagram of the overall result.

**Figure 4:** Influence analysis result of multiple regression.

**Table 1:** The comparison of physical fitness level and fitness consciousness guidance level of investigators.

Group	Before the COVID-19 pandemic appeared			After the COVID-19 pandemic appeared,		
	Physical fitness level (%)	Guidance level of fitness awareness (%)	Exercise frequency (%)	Physical fitness level (%)	Guidance level of fitness awareness (%)	Exercise frequency (%)
Implement physical fitness	56.33 ± 5.21	12.61 ± 6.42	23.34 ± 5.27	88.71 ± 6.22∗	186.49 ± 11.24∗	120.13 ± 9.82∗
Physical fitness has not been implemented	57.84 ± 5.62	12.97 ± 6.53	23.52 ± 5.42	67.42 ± 6.97∗	159.14 ± 7.27∗	103.62 ± 8.14∗
*T*	0.907	0.176	0.107	10.192	9.137	5.239
*P*	0.3703	0.8612	0.9164	0.0003	0.0002	0.0002

Note: Compared with that before implementation, ∗*P* < 0.05.

**Table 2:** The Comparison of exercise frequency, physical injury, and value influence range.

	Exercise frequency		Physical injury		Value influence range	
	Weekly	Monthly	Timely treatment	Simple treatment	Significant impact	Small impact
Before the COVID-19 pandemic appeared (*n* = 20)	18	2	16	4	18	2
After the COVID-19 pandemic appeared (*n* = 20)	12	8	10	10	11	9
*X* ^2^	4.800		3.956		6.144	
*P*	0.0293		0.0472		0.0131	

**Table 3:** Evaluation elements with significant differences.

Factors that differ	Assignment	Remarks
Physical fitness level (%)	<*F* = 0, >*F* = 1	Mainly physical fitness, endurance, strength, and other indicators of exercisers
Guidance level of fitness awareness (%)	<*F* = 0, >*F* = 1	Exercise awareness, fitness awareness, etc.
Exercise frequency (%)	<*c* = 0, >*c* = 1	Weekly frequency, daily frequency
Physical injury (%)	<50 = 0, >50 = 1	Joints, muscles, psychology
Value influence range	>*T* = 0, <*T* = 1	Self-worth, social value

**Table 4:** Influence analysis of multiple regression of influence value.

Correlation evaluation	*B*	*Standard deviation*	*Wald*	*OR*	*P*
Physical fitness level (%)	12.512	5.152	2.612	2.121	0.0001
Guidance level of fitness awareness (%)	2.785	2.372	6.263	2.822	0.3022
Exercise frequency (%)	10.410	4.105	8.821	2.232	0.0001
Physical injury (%)	8.317	12.271	1.122	2.133	0.0002
Value influence range	7.426	9.447	1.627	2.823	0.0003

## Data Availability

The data used to support the findings of this study are available from the corresponding author upon request.
